# Probucol plus cilostazol attenuate hypercholesterolemia-induced exacerbation in ischemic brain injury via anti-inflammatory effects

**DOI:** 10.3892/ijmm.2014.1848

**Published:** 2014-07-10

**Authors:** JI HYUN KIM, KI WHAN HONG, SUN SIK BAE, YONG-IL SHIN, BYUNG TAE CHOI, HWA KYOUNG SHIN

**Affiliations:** 1 Division of Meridian and Structural Medicine, School of Korean Medicine, Pusan National University, Yangsan, Gyeongnam 626-870, Republic of Korea; 2 Department of Pharmacology, School of Medicine, Pusan National University, Yangsan, Gyeongnam 626-870, Republic of Korea; 3 Department of Rehabilitation Medicine, School of Medicine, Pusan National University, Yangsan, Gyeongnam 626-870, Republic of Korea

**Keywords:** cilostazol, focal cerebral ischemia, hypercholesterolemia, inflammatory chemokine, microglia, neuroinflammation, probucol

## Abstract

Probucol, a lipid-lowering agent with anti-oxidant properties, is involved in protection against atherosclerosis, while cilostazol, an antiplatelet agent, has diverse neuroprotective properties. In this study, we investigated the anti-inflammatory effects of probucol and cilostazol on focal cerebral ischemia with hypercholesterolemia. Apolipoprotein E (ApoE) knockout (KO) mice were fed a high-fat diet (HFD) with or without 0.3% probucol and/or 0.2% cilostazol for 10 weeks. To assess the protective effects of the combined therapy of probucol and cilostazol on ischemic injury, the mice received 40 min of middle cerebral artery occlusion (MCAO). Infarct volumes, neurobehavioral deficits and neuroinflammatory mediators were subsequently evaluated 48 h after reperfusion. Probucol alone and probucol plus cilostazol significantly decreased total- and low-density lipoprotein (LDL)-cholesterol in ApoE KO with HFD. MCAO resulted in significantly larger infarct volumes in ApoE KO mice provided with HFD compared to those fed a regular diet, although these volumes were significantly reduced in the probucol plus cilostazol group. Consistent with a smaller infarct size, probucol alone and the combined treatment of probucol and cilostazol improved neurological and motor function. In addition, probucol alone and probucol plus cilostazol decreased MCP-1 expression and CD11b and GFAP immunoreactivity in the ischemic cortex. These findings suggested that the inhibitory effects of probucol plus cilostazol in MCP-1 expression in the ischemic brain with hypercholesterolemia allowed the identification of one of the mechanisms responsible for anti-inflammatory action. Probucol plus cilostazol may therefore serve as a therapeutic strategy for reducing the impact of stroke in hypercholesterolemic subjects.

## Introduction

Hypercholesterolemia is a major underlying cause of ischemic stroke (1) and therapeutics targeting hypercholesterolemia decrease the risk of stroke in high-risk individuals. Chronic systemic inflammatory conditions, such as atherosclerosis, diabetes and obesity are associated with increased risk of stroke (2,3). Stroke is also characterized by massive inflammation in areas surrounding the injury that magnifies damage to the brain (4). Therefore, modulation of inflammation may be an effective therapeutic strategy for reducing the impact of stroke in hypercholesterolemic subjects.

Probucol is a cholesterol-lowering drug with antioxidant, anti-inflammatory and anti-atherosclerogenic properties (5). Cilostazol is a type 3 phosphodiesterase inhibitor that exhibits antiplatelet and vasodilating activity by suppressing the degradation of cAMP (6). Cilostazol has also been shown to exert *in vivo* neuroprotective effects against cerebral ischemic injury via anti-inflammatory effects (7). A previous *in vitro* study using cultured human coronary artery endothelial cells (8), as well as *in vivo* studies in rats, low-density lipoprotein (LDL) receptor-deficient mice and apolipoprotein E (ApoE) knockout (KO) mice revealed the synergistic effects of probucol plus cilostazol against atherosclerotic lesions and ischemic brain injury (9–11). The aforementioned studies suggested that combined administration of these drugs may result in synergistic effects in mice with stroke and hypercholesterolemia. In addition, probucol and cilostazol have anti-inflammatory effects and may act synergistically to accelerate the outcome process via the inhibition of inflammation.

Chemokines, which are well-known regulators of peripheral immune cell recruitment and trafficking under physiological and pathological conditions, can cause secondary damage during inflammation and affect cerebral ischemia. MCP-1, a pro-inflammatory chemokine, is a potent chemoattractant capable of promoting monocyte recruitment into an inflammatory or pathological site. Once activated near the site of pathology, the recruited cells can produce more pro-inflammatory mediators, inducing inflammation (12,13). Therefore, understanding the modulation of chemokines may result in the development of treatments specific for cerebral ischemia with hypercholesterolemia.

In the present study, we investigated whether hypercholesterolemia exacerbates ischemic outcomes and any exacerbation of stroke was associated with neuroinflammation in the brain by coupling hypercholesterolemia in an experimental stroke model using mice. In addition, we focused on the effect of probucol and cilostazol administered in combination with conventional therapy due to their anti-inflammatory properties. The tissue outcome and functional outcome were determined following transient middle cerebral artery occlusion (MCAO) in ApoE KO mice fed the high-fat diet (HFD) for 10 weeks using combinatorial treatment of probucol plus cilostazol. Microglia and astrocyte activation in accordance with chemokine levels were determined to be the action mechanisms. The current study presented evidence with regard to the anti-inflammatory effects of combinatorial therapy with probucol and cilostazol during the management of stroke patients undergoing hypercholesterolemia.

## Materials and methods

### General surgical preparation

Male ApoE KO mice (Japan SLC, Shizuoka, Japan) with a C57BL/6J genetic background were housed under diurnal lighting conditions and allowed food and tap water *ad libitum*. The study was carried out in strict accordance with the recommendations in the Guide for the Care and Use of Laboratory Animals of the National Institutes of Health. In addition, the protocol was approved by the Pusan National University Institutional Animal Care and Use Committee (permit no.: PNU-2011-000419). Four-week-old ApoE KO mice were fed a Western-type HFD (42% of total calories from fat, 0.15% cholesterol; Research Diets, Inc., New Brunswick, NJ, USA) containing 0.3% (wt/wt) probucol, 0.2% (wt/wt) cilostazol, or 0.3% (wt/wt) probucol and 0.2% (wt/wt) cilostazol for 10 weeks. Anesthesia was achieved by isoflurane (2% induction and 1.5% maintenance, in 80% N_2_O and 20% O_2_) administered via a face mask. The femoral artery was catheterized for measurement of the mean arterial blood pressure using a model MLT844 physiological pressure transducer (AD Instruments, Medford, MA, USA). The data were continuously recorded using a Power Lab data acquisition and analysis system (AD Instruments) and stored in a computer. The depth of anesthesia was checked by the absence of cardiovascular changes in response to tail pinch. Rectal temperature was kept at 36.5–37.5°C using a Panlab^TM^ thermostatically controlled heating mat (Harvard Apparatus, Holliston, MA, USA). Arterial blood gases and pH were measured prior to ischemia using i-Stat System (Abbott, Abbott Park, IL, USA).

### Focal cerebral ischemia

A fiber-optic probe was affixed to the skull over the MCA for measurement of the regional CBF (rCBF) by a PeriFlux Laser Doppler System 5000 (Perimed, Stockholm, Sweden). Baseline values were measured prior to internal carotid artery ligation (considered to be 100% flow). Focal cerebral ischemia was induced by occluding the MCA using a previously described intraluminal filament technique (14). MCAO was induced by a silicon-coated 7-0 monofilament in the internal carotid artery and the monofilament was advanced to occlude the MCA. In all the animals, rCBF was measured to confirm the achievement of consistent and similar levels of ischemic induction. The filament was withdrawn 40 min after occlusion and reperfusion was confirmed using laser Doppler. The surgical wound was sutured and mice were allowed to recover from anesthesia. The brains were removed at 48 h after MCAO. Cerebral infarct size was determined on 2,3,5-triphenyltetrazolium chloride (TTC)-stained, 2-mm-thick brain sections (n=10–11). Infarction areas were quantified with iSolution full image analysis software (Image & Microscope Technology, Vancouver, BC, Canada). To account for and eliminate the effects of swelling/edema, infarction volume was calculated by indirect measurement by summing the volumes of each section according to the formula: contralateral hemisphere (mm^3^) - undamaged ipsilateral hemisphere (mm^3^) (15).

### Neurological score

Neurological deficit was scored in each mouse at 24 and 48 h after ischemic insult in a blinded manner according to the following graded scoring system (n=12–14): 0, no deficit; 1, forelimb weakness and torso turning to the ipsilateral side when held by tail; 2, circling to the affected side; 3, unable to bear weight on the affected side; and 4, no spontaneous locomotor activity or barrel rolling (16).

### Wire-grip test

Vestibule-motor function was assessed using a wire-grip test 24 and 48 h after cerebral ischemia (17) (n=12–14). Briefly, mice were placed on a metal wire (45 cm long) suspended 45 cm above protective padding and allowed to traverse the wire for 60 sec. The latency for which a mouse remained on the wire within a 60-sec interval was measured, and the wire grip score was quantified using the following 5-point scale: unable to remain on the wire for 30 sec, 0; failure to hold on to the wire with both sets of fore paws and hind paws together, 1; holding on to the wire with both forepaws and hind paws but not the tail, 2; holding on to the wire using the tail along with both forepaws and both hind paws, 3; moving along the wire on all four paws plus tail, 4; a score of 4 points in addition to the mouse ambulating down one of the posts used to support the wire, 5. Tests were administered in triplicate and the average value was calculated for each mouse on each test day.

### Cylinder test

The cylinder test was modified for mice in order to determine forelimb use and rotation asymmetry (18) (n=12–14). Briefly, the mouse was placed in a transparent cylinder (diameter, 9-cm and height, 15 cm). After the mouse was placed into the cylinder, forelimb use of the first contact against the wall following rearing and during lateral exploration was recorded. The final score was calculated as: (non-impaired forelimb movement - impaired forelimb movement)/(non-impaired forelimb movement + impaired forelimb movement + both movement). This test evaluates forelimb use asymmetry for weight shifting during vertical exploration and provides high inter-rater reliability, even when inexperienced raters are included.

### Isolation of total RNA and RT-PCR

Total RNA was isolated from the ischemic area in the brain using TRIzol (Invitrogen Life Technologies, Carlsbad, CA, USA) according to the manufacturer’s insructions (n=5). The total RNA was reverse-transcribed for 1 h at 42°C with Moloney Murine Leukemia Virus reverse transcriptase (Promega, Madison, WI, USA) to produce cDNA. RT-generated cDNA encoding the *MCP-1*, *VCAM*, *iNOS*, *COX-2*, *TNF-α*, *IL-1β* and *GAPDH* genes was amplified by PCR using the primers: MCP-1 (forward 5′-TGGCTCAGCCAGA TGCAGTTAA-3′ and reverse 5′-CTAGTTCACTGTCACAC TGGTC-3′), VCAM (forward 5′-GAACCTGACCTGCTCAA GTGAT-3′ and reverse 5′-TACCAAGGAAGATGCGCAG TAG-3′), iNOS (forward 5′-CACTTGGATCAGGAACCTG AAG-3′ and reverse 5′-CCAGCTTCTTCAATGTGGTAGC-3′), COX-2 (forward 5′-CTTGGTCTACAAGACGCCACAT-3′ and reverse 5′-GCCATAGAATAATCCTGGTCGG-3′), TNF-α (forward 5′-CATCTTCTCAAAATTCGAGTGACAA-3′ and reverse 5′-TGGGAGTAGACAAGGTACACCCC-3′), IL-1β (forward 5′-AAGGGCTGCTTCCAAACCTTTGAC-3′ and reverse 5′-TGCCTGAAGCTCTTGTTGATGTGC-3′) and mGAPDH (forward 5′-ATGACCACAGTCCATGCCATCA-3′ and reverse 5′-TTACTCCTTGGAGGCCATGTAG-3′). Products were size-separated by electrophoresis on 2% agarose gels and visualized after staining with ethidium bromide. Thermal cycling conditions consisted of 94°C for 5 min and 30 cycles of 94°C for 30 sec, 55°C for 30 sec and 72°C for 30 sec.

### Immunohistochemistry

Forty-eight hours after MCAO, the mice were deeply anesthetized with thiopental sodium and subsequently perfused transcardially with cold phosphate buffered saline (PBS), after which they were perfused for fixing using 4% paraformaldehyde (n=3). The brain of each mouse was then removed and fixed for 48 h in 4% paraformaldehyde at 4°C. Subsequently, it was subjected to cryoprotection in 30% sucrose for 24 h at 4°C. The isolated brains were then frozen and stored at −80°C until further processing. The frozen brains were cut into sections (14 μm) using a model CM 3050 cryostat (Leica Microsystems, Wetzlar, Germany). The sections were immunostained with antibodies against MCP-1 (Abcam, Cambridge, UK), CD11b (Serotec, Oxford, UK) and GFAP (Dako, Glostrup, Denmark). After additional incubation with biotinylated secondary antibody, the samples were incubated in ABC reagent (Vector Laboratories, Burlingame, CA, USA). Reactions were visualized by development in 3,3′-diaminobenzidine substrates (Vector Laboratories). The samples were then visualized using a light microscope (Carl Zeiss, Jena, Germany).

### Drugs

Probucol [4,4′-(isopropylidenedithio)bis(2,6-di-t-buty- lophenol)] and cilostazol [OPC-13013, 6-[4-(1-cycl ohexyl-1H -tetrazol-5-yl) butoxy]-3,4-dihydro-2-(1H)-quinolinone] were donated by Otsuka Pharmaceutical (Tokushima, Japan) and were added to the HFD.

### Data analysis

Data are expressed as the means ± standard error of the mean (SEM). The control vs. vehicle group and vehicle vs. probucol-treated group were compared by the unpaired t-test, while vehicle vs. each concentration of probucol was compared by one-way ANOVA followed by Dunnett’s test. Differences were considered statistically significant, when the two-tailed P-values were <0.05. Statistical analyses were performed using the SAS software (SAS Institute Japan, R9.1).

## Results

### Physiological parameters

The body weights of ApoE KO mice fed a HFD for 10 weeks were higher than those of mice fed a normal diet (control) (32.71±1.05 vs. 25.90±0.73 g, respectively, P<0.01; n=15–16). Treatment with 0.3% probucol and 0.2% cilostazol did not affect the body weight or blood pressure of HFD-fed mice (Table I). After 10 weeks of HFD, large increases in total cholesterol and LDL-cholesterol plasma were observed in ApoE KO mice (P<0.01 vs. control) (Table I). Probucol alone and probucol plus cilostazol in combination led to a significant decrease in the total- and LDL-cholesterol levels in ApoE KO mice fed the HFD (P<0.01 vs. vehicle).

### Effect of probucol plus cilostazol in combination on tissue and functional outcome in focal cerebral ischemia

To determine whether probucol plus cilostazol improved the tissue outcome after cerebral ischemia in hypercholesterolemic mice, the infarct size was measured 48 h after a 40-min transient MCAO. MCAO resulted in 137% larger infarct volumes in ApoE KO fed the HFD for 10 weeks when compared to those fed the regular diet (47.66±10.15 mm^3^ vs. 20.13±4.76 mm^3^; P<0.05) (Fig. 1A and B); however, this increase was significantly reduced by treatment with probucol plus cilostazol (20.90±3.71 mm^3^; P<0.05 vs. vehicle group). The group that received probucol alone also tended to have a smaller infarct volume (22.79±3.93 mm^3^; P=0.055 vs. vehicle group). To assess the effects of probucol plus cilostazol on functional recovery after cerebral ischemia in hypercholesterolemic mice, the neurological score, wire-grip test and cylinder test were assessed 24 and 48 h after a 40-min transient MCA occlusion. Consistent with a smaller infarct size, probucol alone and combined treatment with cilostazol led to prominent improvement of neurological and motor function at both 24 and 48 h after ischemic injury (Figs. 1C and 2).

### Effect of probucol plus cilostazol in combination on inflammatory mediator mRNA levels in the ischemic brain

To examine the anti-neuroinflammatory effects of probucol plus cilostazol on focal cerebral ischemia with hypercholesterolemia, we assessed the mRNA levels of MCP-1, VCAM, iNOS, COX-2, TNF-α and IL-1β in the ischemic brain. MCP-1, iNOS, TNF-α and IL-1β mRNA levels were increased in the ischemic brain of hypercholesterolemic mice, but VCAM and COX-2 mRNA levels were not increased. Moreover, this increase of MCP-1 and TNF-α mRNA was significantly decreased by probucol plus cilostazol in combination compared with the vehicle group (Fig. 3).

### Effect of probucol plus cilostazol in combination on MCP-1, CD11b and GFAP expression in the ischemic cortex

MCP-1 expression in the ischemic brain was assessed by immunohistochemistry. MCP-1 expression increased in the ischemic brain of hypercholesterolemic mice, which was decreased by probucol alone, cilostazol alone or probucol plus cilostazol (Fig. 4A). CD11b (also known as α_m_β_2_ integrin and Mac1) and GFAP are sensitive markers of microglial and astrocyte activation, respectively. CD11b immunoreactivity was increased in the vehicle group, but this increase was attenuated by probucol alone and probucol plus cilostazol (Fig. 4B). Immunostaining of GFAP was evident in the ischemic brain of the control and hypercholesterolemic mice and mild GFAP immunostaining appeared in mice that received probucol alone, cilostazol alone and probucol plus cilostazol (Fig. 4C).

## Discussion

The present study was conducted to elucidate the protective effects of probucol plus cilostazol in combination against cerebral ischemic injury with hypercholesterolemia and the mechanism by which these effects occur. MCAO (40 min) and reperfusion (48 h) resulted in significantly larger infarct volumes in ApoE KO mice fed HFD for 10 weeks when compared to ApoE KO mice fed a regular diet, although these increased volumes were significantly reduced in the probucol plus cilostazol group. Consistent with the smaller infarct size, probucol alone and combined treatment with cilostazol greatly improved the neurological and motor function. In addition, probucol alone and probucol and cilostazol in combination decreased MCP-1 mRNA expression, as well as MCP-1, CD11b and GFAP immunoreactivity in the ischemic cortex. These findings suggest that the inhibitory effect of probucol and cilostazol in combination through an inflammatory mediator, MCP-1 expression, in the ischemic brain with hypercholesterolemia allowed the identification of one of the mechanisms responsible for its anti-inflammatory action.

The lack of successful translation from the laboratory to clinical settings may be the result of prevailing clinical conditions, such as hypercholesterolemia, hypertension and insulin intolerance, which are correlated with a higher incidence of stroke (2,19,20), which are not included in animal models used in the study of stroke. Animal stroke studies conducted using mostly young animals without risk factors (21) do not accuratley reflect the pathophysiological conditions in humans. The ApoE KO mouse model is the classical model of atherosclerosis. These mice start to develop severe hypercholesterolemia, induce inflammation and atherosclerotic lesions in the aorta and pulmonary, coronary and carotid arteries at the age of 8 or 10 weeks, depending on the type of diet administered (22). By coupling hypercholesterolemia in an experimental mouse stroke model, the present study investigated whether hypercholesterolemia exacerbates ischemic outcomes and any exacerbation of stroke was connected with inflammation in the brain. In addition, we addressed whether probucol and cilostazol administered in combination attenuate hypercholesterolemia-induced exacerbation in ischemic brain injury via anti-inflammatory effects.

Hypercholesterolemia is a risk factor for ischemic stroke. In large clinical trials or patient registries, ~45–60% of patients exhibit elevated serum cholesterol levels (23,24). It is well known that cholesterol induces inflammation in the brain (25–27), and that oxidized metabolites of cholesterol may be involved in the upregulation of inflammatory markers (28,29). There is also considerable evidence that hypercholesterolemia and derivations of cholesterol contribute to a breakdown of the blood brain barrier (30,31), thereby making hypercholesterolemic patients more susceptible to stroke. Consistent with the aforementioned studies, our results showed that ischemic cerebral infarcts induced by 40 min MCAO and 48 h reperfusion resulted in significantly larger infarct volumes, neurological deficits and motor deficits in ApoE KO mice fed HFD for 10 weeks when compared to ApoE KO mice fed a regular diet. These results are similar to those of a previous study (11). Moreover, MCP-1 mRNA levels and MCP-1, CD11b and GFAP immunoreactivity, which are thought to be involved in neuroinflammation, increased in the ischemic brain of hypercholesterolemic mice.

Obesity is also a well-established major risk factor for stroke (32). Clinical studies suggest that the prevalence of ischemic stroke has markedly increased in children and young adults, which positively correlated with an increase in risk factors including obesity, lipid disorders and diabetes (33). In addition, experimental studies in genetic or diet-induced obesity models have shown increased cerebral infarct size and poor outcomes of stroke (34,35). In the present study, we found that the body weights of ApoE KO mice fed a HFD for 10 weeks were significantly higher than those of mice fed a regular diet. However, although probucol alone and probucol plus cilostazol in combination did not affect the body weight, they improved tissue and functional outcome after ischemic brain injury with hypercholesterolemia. On the other hand, probucol alone and probucol plus cilostazol in combination led to a significant decrease in total- and LDL-cholesterol levels in ApoE KO mice fed the HFD, suggesting that the beneficial effects of probucol and cilostazol in stroke with hypercholesterolemia may be due, not to lowering body weight, but only in part to lipid-lowering properties of the drugs.

Inflammation in the brain caused by activated microglia is a prominent pathological feature associated with hypercholesterolemia or ischemic stroke. Under pathological conditions, activated microglia release a variety of neurotoxic compounds and proinflammatory mediators, which are thought to be responsible for the pathological conditions. MCP-1 is a particularly important chemokine that is primarily responsible for the initiation and progression of inflammatory responses by promoting the migration and recruitment of inflammatory cells (36). MCP-1 has been found to regulate the migration of activated microglia cells to sites of inflammation in the CNS (37). Overexpression of MCP-1 exacerbates ischemic injury and enhances recruitment of inflammatory cells to the sites of injury (38), whereas absence of the *mcp-1* gene has been shown to reduce ischemia-reperfusion injury (39). We found increased MCP-1, CD11b and GFAP immunoreactivity in hypercholesterolemic ischemic brains, suggesting that MCP-1 production and microglia and astrocyte activation are involved in the promotion of hyperlipidemia-induced inflammation and injury in the ischemic brain. Profound shifts to the reduced MCP-1 and microglia and astrocyte activation in probucol plus cilostazol-treated mice suggest that probucol and cilostazol in combination exert neuroprotective effects via anti-inflammation in hypercholesterolemic ischemic brains.

Probucol, a lipid-lowering agent with antioxidant properties, is involved in the protection against atherogenesis (40). Probucol is capable of inhibiting the expression of oxidation-sensitive inflammatory factors, such as VCAM-1 (41), MCP-1 (42) and IL-1 (43), and attenuating inflammation and increasing stability of vulnerable atherosclerotic plaques in rabbits (44). Serum concentrations of inflammatory cytokines and matrix metalloproteinases, and expression levels of the Toll-like receptor (TLR)-2, TLR-4, MCP-1, ICAM-1, scavenger receptor A, CD36 and oxidized LDL receptor 1 within the lesions were markedly decreased in probucol treatment groups as compared to the control group (44). Cilostazol, another drug in the combination treatment in this study, is an inhibitor of type 3 phosphodiesterase that exerts antiplatelet activity through the suppression of cAMP degradation (6) and also has pleiotropic effects against inflammation on vascular function and atherosclerosis (45). Furthermore, cilostazol has demonstrated *in vivo* neuroprotective effects against cerebral ischemic injury via anti-inflammatory effects (7). Therefore, the combination of probucol and cilostazol may have a synergistic effect, as the two agents inhibit inflammation. A previous *in vitro* study of cultured human coronary artery endothelial cells (8), *in vivo* studies in rats, LDL receptor-deficient mice and ApoE KO mice revealed a synergistic effect of probucol plus cilostazol against atherosclerotic lesions and ischemic brain injury (9–11). Park *et al* showed that probucol and cilostazol combination therapy inhibited the expression of VCAM-1 and MCP-1 in cultured human coronary artery endothelial cells with MCP-1 being more effectively inhibited than when treated with probucol or cilostazol monotreatment (8).

Recently, authors of this study demonstrated a cerebrovascular protective effect of probucol plus cilostazol in combination in focal ischemic mice with hypercholesterolemia that occurred via the upregulation of endothelial nitric oxide synthase and adiponectin in acute ischemic injury (11). In the present study, we focused on the inflammatory properties of probucol and cilostazol administered in combination with conventional therapy in the subacute phase after cerebral ischemia. In addition, we reduced the probucol dose from 0.5 to 0.3% to observe the synergistic effects of probucol and cilostazol against cerebral ischemic brain injury with hypercholesterolemia in this study. Treatment with 0.3% probucol plus 0.2% cilostazol significantly reduced the infarct volume with, not only neurological deficits, but also motor deficits in ApoE KO mice fed a HFD. Furthermore, probucol and cilostazol in combination reduced hyperlipidemia-induced inflammation via the inhibition of MCP-1 and microglia and astrocyte activation. However, 0.3% probucol is likely too high a dose for the synergistic effects of probucol and cilostazol to become evident. Accordingly, more studies are required to determine the clinically relevant probucol dose for the synergistic effect of probucol and cilostazol in ischemic brain injury with hypercholesterolemia. Collectively, the beneficial effects of probucol and cilostazol in stroke with hypercholesterolemia may be due only in part to lipid-lowering properties, with the primary benefit derived from improved endothelial function and the anti-inflammatory actions of the drugs.

In summary, the present study has demonstrated that probucol and cilostazol in combination exerted inhibitory effects against the expression of the inflammatory chemokine, MCP-1, in ischemic brains with hypercholesterolemia, which allowed identification of one of the mechanisms responsible for its anti-inflammatory action. These findings suggest that probucol plus cilostazol is a potential therapeutic strategy for reducing the impact of stroke in hypercholesterolemic subjects.

## Figures and Tables

**Figure 1:** Effect of probucol plus cilostazol in combination on infarct volume and neurological deficit in cerebral ischemic mice with hypercholesterolemia. (A) Representative images of 2,3,5-triphenyltetrazolium chloride (TTC)-stained brains from apolipoprotein E (ApoE) knockout (KO) mice fed a high-fat diet (HFD) with or without 0.3% probucol (Pro), 0.2% cilostazol (Cilo) or 0.3% probucol plus 0.2% cilostazol for 10 weeks. Mice were subjected to 40 min MCA occlusion followed by 48 h reperfusion. White indicates the infarct area. (B) Quantification of infarct volume at 48 h after ischemia (n=10–11). Infarct volume was calculated by integrating the infarct area in 2 mm-thick coronal slices. (C) Neurological deficit was assessed in each mouse at 24 and 48 h after ischemic insult in a blinded manner (n=12–14). Values are the mean ± standard error of the mean (SEM). ^*^P<0.05 vs. age-matched ApoE KO mice without HFD [Con (control)]; ^#^P<0.05 and ^##^P<0.01 vs. age- and diet-matched ApoE KO mice [Veh (vehicle)].

**Figure 2:** Effect of probucol plus cilostazol in combination on motor functional outcome in cerebral ischemic mice with hypercholesterolemia. (A) Vestibule-motor function was assessed by a wire grip test and (B) asymmetric forelimb use for weight shifting by a cylinder test. Values are the mean ± standard error of the mean (SEM). ^**^P<0.01 vs. age-matched apolipoprotein E (ApoE) knockout (KO) without high-fat diet (HFD) [Con (control)]; ^#^P<0.05 and ^##^P<0.01 vs. age- and diet-matched ApoE KO mice [Veh (vehicle)].

**Figure 3:** Effect of probucol plus cilostazol in combination on inflammatory mediator mRNA levels in the ischemic brain. (A) Representative PCR products in the ischemic brain 48 h after MCAO. (B) Densitometric analysis of the PCR band. Relative abundance of MCP-1, VCAM, iNOS, COX-2, TNF-α and IL-1β compared with GAPDH. The results are expressed as the mean ± standard error of the mean (SEM) (n=5). ^**^P<0.01 vs. age-matched apolipoprotein E (ApoE) knockout (KO) mice without high-fat diet (HFD) [Con (control)]; ^#^P<0.05 and ^##^P<0.01 vs. age- and diet-matched ApoE KO mice [Veh (vehicle)].

**Figure 4:** Effect of probucol plus cilostazol in combination on MCP-1 expression and microglia and astrocyte activation in the ischemic brain. Apolipoprotein E (ApoE) knockout (KO) mice were fed a high-fat diet (HFD) with or without 0.3% probucol (Pro), 0.2% cilostazol (Cilo), or both (Pro+Cilo) for 10 weeks. Coronal sections of ischemic brain 48 h after MCA occlusion were stained immunohistochemically with (A) MCP-1, (B) CD11b, a sensitive marker of microglial activation, and (C) GFAP antibody, a sensitive marker of astrocyte activation. The blue rectangle represents the imaging field. MCP-1, CD11b and GFAP immunoreactivity was increased in the vehicle group, but was attenuated by treatment with probucol and cilostazol in combination. Scale bar, 10 μm.

**Table I:** Physiological parameters.

Variables	Control (n=15)	Vehicle (n=16)	Probucol (n=15)	Cilostazol (n=15)	Probucol + cilostazol (n=16)
Body weight	25.90±0.73	32.71±1.05^b^	33.77±0.51	33.99±1.25	33.09±0.63
MABP	82.48±2.36	89.38±2.13^a^	85.17±3.09	87.34±1.77	85.34±2.12
pH	7.34±0.01	7.33±0.01	7.32±0.02	7.32±0.01	7.32±0.01
pO_2_	111.13±4.11	105.75±3.56	107.33±3.68	111.20±3.34	112.94±3.82
pCO_2_	41.56±1.62	38.76±1.21	41.05±1.68	33.38±1.40	39.67±0.20
Total cholesterol	261.67±5.24	546.33±33.05^b^	245.00±14.47^c^	531.67±16.29	242.00±13.05^c^
LDL-cholesterol	211.67±3.53	420.67±28.72^b^	185.67±18.77^c^	409.33±20.85	179.00±5.57^c^

Values are the mean ± SEM. Body weight is expressed in grams. MABP, pO_2_ and pCO_2_ are expressed in mmHg.

a P<0.05 and

b P<0.01 vs. age-matched ApoE KO without HFD (control);

c P<0.01 vs. age- and diet-matched ApoE KO (vehicle).

MABP, mean arterial blood pressure; LDL, low-density lipoprotein; SEM, standard error of the mean; ApoE, apolipoprotein E; KO, knockout; HFD, high-fat diet.
